# Application of Surface-Enhanced Raman Spectroscopy in the Screening of Pulmonary Adenocarcinoma Nodules

**DOI:** 10.1155/2022/4368928

**Published:** 2022-06-23

**Authors:** Bowen Peng, Huan Yan, Runrui Lin, Gang Yin

**Affiliations:** ^1^Nanjing University, School of Electronic Science and Engineering, Nanjing 210023, China; ^2^School of Medicine, University of Electronic Science and Technology of China, Chengdu 611731, China; ^3^Sichuan Cancer Hospital & Institute, Radiation Oncology Key Laboratory of Sichuan Province, Chengdu 610041, China

## Abstract

This study is aimed at evaluating the feasibility of a screening method for the pulmonary adenocarcinoma nodules through surface-enhanced Raman spectroscopy (SERS). *Objective*. Using SERS to measure serum from pulmonary nodules and healthy subjects, intraoperative biopsy pathological diagnosis was regarded as the gold standard for labeling serum samples. To explore the application value of SERS in the differential diagnosis of pulmonary adenocarcinoma nodules, benign nodules, and healthy, we build a machine learning model. *Method*. We collected 116 serum samples from patients. Radiographically confirmed nodules less than 3 cm in maximum diameter in all patients, including 58 cancer (pathologic diagnosis: adenocarcinoma nodules, labeled as cancer) patients, 58 pathologic diagnoses as benign nodule (labeled as benign) patients, and 63 healthy (labeled as normal) people from the clinical laboratory of Sichuan Cancer Hospital. Gold nanorods were employed as SERS substrates. Support vector machine (SVM) was used to classify the normal, benign, and cancer sample groups, and SVM model evaluated using cross-validation. *Results*. The average SERS spectra of serum were significantly different between the normal group and the cancer/benign group. While the average SERS spectra of the cancer group and the benign group differed slightly, for the cancer, benign, and normal groups, SVM models can predict with 93.33% accuracy. *Conclusion*. This exploratory study demonstrates that the SERS technique based on nanoparticles in conjunction with SVM has great potential as a clinical auxiliary diagnosis and screening for pulmonary adenocarcinoma nodules.

## 1. Introduction

Lung cancer is the leading cause of cancer deaths globally, and the mortality rates of lung cancer occupy the first position among all cancers. It is estimated that there are 2.09 million new cases and 1.76 million deaths from lung cancer worldwide each year [1]. And the overall 5-year survival rate in lung cancer patients was only 18.7% in China [2]. However, the corresponding operation of radiotherapy and chemotherapy intervention for lung cancer of diagnosis in the early stage can improve patients' survival rate [3]. Currently, the primary screening method for early lung cancer is low-dose CT (LDCT) [4]. Early stage of lung cancer is mainly manifested in pulmonary nodules; CT may detect the early small pulmonary nodules, but it contains radiation risk [5]. Moreover, exposure to ionizing radiation should be avoided in certain groups, such as the elderly, women planning pregnancy, pregnant and lactating mothers, and people with thyroid problems. In addition, there are other methods for early-stage lung cancer screening using circulating or noncirculating markers [6]. The marker detection method is a body fluid-based analysis method, including circulating tumor cell detection and biomarker detection [7]. However, the low concentration and low correlation of specific markers also make it difficult for these liquid biopsies to obtain significant indicative results, and the price is relatively high. Therefore, there is a great need to explore simple, reliable, and low-cost methods to diagnose benign and malignant pulmonary nodules.

Through the continuous development of imaging examination methods, the necessary interventions such as surgical resection and radiofrequency ablation in the early stage of lung cancer patients can improve their survival rate and quality of life significantly and even achieve an effectiveness of the cure. Bronchoscopy and CT-guided biopsy can provide an accurate pathological diagnosis. However, adenocarcinoma frequently occurs in subsegmental bronchi or alveoli, which are often inaccessible by bronchoscopy. The pathological results are always difficult to obtain. Also, CT-guided puncture biopsy is invasive, and some patients cannot tolerate it. CT is also affected by the degree of cooperation of patients and the operator's technical level. Presently, the discovery and diagnosis of pulmonary nodules mainly rely on CT examination. For the patient who cannot take a puncture biopsy, the diagnosis of pulmonary nodules still needs an intraoperative pathological biopsy. Adenocarcinoma is the primary pathological type of malignant pulmonary nodules. To improve the accuracy of preoperative diagnosis and early diagnosis, it is necessary to reduce unnecessary intervention for patients with benign nodules, particularly invasive surgery, and to develop radiation-free, low-injury, low-cost, and easily popularized approaches [8, 9].

Raman spectroscopy is an analytical method for studying molecular structure by analyzing the scattering spectra of target molecules by extracting information on molecular vibration and rotation. And the Raman characteristic spectrum of early cancer tissue and body fluid is different from that of normal tissue, making Raman spectroscopy a promising candidate for early cancer screening.

On the other hand, both markers and metabolites may face deficient levels in the early stage of tumor formation [10, 11]; it is necessary to effectively amplify the Raman signal for effective observation in the practical phase. Surface-enhanced Raman spectroscopy (SERS) is an enhancement effect on the surface of nanosized metal structures, which can escalate the intensity of ordinary Raman scattering by several orders of magnitude, even to the level of single-molecule detection. SERS has the advantages of high sensitivity, fast detection speed, low cost, and strong versatility and has been widely used in many fields such as biomedicine [12], drug detection, and bacterial detection [13]. The serum is composed of water, carbohydrates, proteins, and other components. During the cell carcinogenesis process, the types and contents of substances in serum will change. The Raman signal of many substances is relatively weak, and sometimes, the clinic-pathological symptoms of cancer patients may not be obvious enough to diagnose. By measuring the SERS spectra of biofluids, the characteristics of cancer could be reflected in the spectral difference to provide a reference for the diagnosis of cancer. Pichardo-Molina et al. studied Raman spectroscopy for identifying serum from healthy and breast cancer patients. The multivariate statistical analysis constructed the diagnostic model, obtaining a sensitivity of 97% and a specificity of 78% [14]. Chowdary et al. compared the Raman spectra of normal colon samples and cancerous colon samples (*N* = 11 cases, 102 Raman spectra). They found that the Raman spectra of cancerous tissues were relatively higher than those of normal tissues. It has a larger spectrum, indicating that cancerous tissue has more biological macromolecules than normal tissue, which provides the primary basis for the early diagnosis of colon cancer [15]. The characteristic peaks in the Raman spectrum are referred to as “fingerprints” and represent the biochemical composition of the sample. Raman spectroscopy can be used as an in vitro, minimally invasive, or even noninvasive early cancer detection technology.

This project plans to use precious metal nanoparticles as the SERS substrate. Serum from pulmonary adenocarcinoma patients, benign pulmonary nodules, and healthy patients (control group) was tested and classified by SVM to evaluate their detection ability.

In this study, we used a retrospective research method, with pathological diagnosis as the gold standard to label serum, and collected the surface-enhanced Raman spectroscopy of serum. SVM was used to establish a classification model for analyzing benign and malignant pulmonary nodules, which may be an additional tool for surgery or diagnosing pulmonary adenocarcinoma nodules.

## 2. Methods

### 2.1. Research Object

The Ethics Committee of Sichuan Cancer Hospital approved this study, and all serum data were collected at Sichuan Cancer Hospital from July 1, 2020, to November 31, 2021. Inclusion and exclusion criteria are as follows:

1. Patients with malignant lung tumors: ① the diagnosis of lung cancer (adenocarcinoma) was confirmed by pathology, pulmonary nodules ≤ 3 cm; ② no surgery, radiotherapy, and chemotherapy were received before sample collection; ③ no combined systemic tumors; ④ no other diseases; ⑤ those who have no heart, liver, kidney, and other organ dysfunction; and ⑥ blood routine, liver, and kidney functions are normal
2. Patients with benign lung tumors: ① the pathological diagnosis is benign (inflammation, pulmonary tuberculosis, lung cyst, etc.), pulmonary nodules ≤ 3 cm; ② no history of malignant tumor; ③ no other diseases; ④ no heart, liver, kidney, and other organ dysfunction; and ⑤ blood routine, liver, and kidney function are normal
3. Normal control group: ① no history of malignant tumor; ② no heart, liver, kidney, and other organ dysfunction; ③ normal blood routine, liver, and kidney function; ④ body mass index (BMI) range of 18.5-23.9; and ⑤ no lung nodules nodes and inflammatory lesions

Serum collection: after fasting for 8 hours, the subjects take 2 mL of fasting venous blood at 6-7 o'clock the following day without adding anticoagulants. The upper serum was taken as a sample and frozen in a -80°C refrigerator after centrifugation at 4000 R/min for 10 minutes.

They were selected from 116 patients with pulmonary nodules in Sichuan Cancer Hospital, including 58 cancer (adenocarcinoma nodules, labeled as cancer) patients, 58 benign patients (labeled as benign), and 63 healthy (labeled as normal) people. The mean age of the cancer group is 57.5 ± 9.6, including 34 males and 24 females. The mean age of the benign patient group is 52.4 ± 11.8, including 23 males and 35 females. A total of 63 healthy people (26 males, 34 females, age 60.4 ± 13.7 years old) were selected from the health examination of our hospital as the control group. General information of all investigated individuals, such as gender, age, clinical stage, tumor type, and tumor growth location, is shown in Table 1. All individuals participating in the study gave informed consent and signed informed consent for the study purpose.

### 2.2. Substrate Production

We prepared a freshly mixed solution with 0.01 M sodium borohydride dissolved in 0.01 M sodium hydroxide. Take an HAuCl4 solution (10 mL, 0.5 mM) in 0.1 M CTAB added to 460 *μ*L of the sodium borohydride aqueous solution, and rapidly stir the mix solution, leading to a change in color from greenish to light brown. Silver nitrate (70 *μ*L, 0.1 M) solution was added to an HAuCl4 solution (10 mL, 0.5 mM) in 0.1 M CTAB, followed by the addition of hydroquinone aqueous solution (500 *μ*L, 0.1 M), and the resulting mixture was hand-stirred until it became clear. Next, 160 *μ*L of seed solution was added, and the growth solution was mixed thoroughly and allowed to age overnight [16].  Figure 1 is the transmission electron microscope image of the synthesized gold nanorods.

### 2.3. Test Method

The instrument used is the Horiba iHR550 remote fiber-coupled Raman microscope system. It carries a fiber-coupled microscope that provides complete microscopic analysis capabilities simple and cost-effective manner. The serum of the investigated individuals obtained from the Laboratory Department of the Provincial Cancer Hospital will be stored in a -80°C freezer until subsequent testing. Before starting the test, concentrated sulfuric acid was added to a 30% hydrogen peroxide solution (volume ratio is 7 : 3), and glass slides with a size of 1 cm × 1 cm were soaked in the solution for 1 minute. The slides were then washed with deionized water and dried to ensure cleanness. The serum to be tested and the gold nanorods were mixed at a ratio of 1 : 1, mixed evenly with a pipette, and dried at room temperature for 30 min. Then, a drop of the hybrid solution was placed on the cleaned glass slide for SERS detection. Each sample measures 8 spectra at different positions. The experiment was carried out in a dark room, all operated by the same person. Spectral calibration of the Horiba iHR550 using a single crystal silicon wafer (which continuously emits a characteristic peak at 520.7 cm^−1^) is required before sampling. After calibration, the SERS measurement was performed with an incident laser at 785 nm, whose power was 5 mW. The accumulation time of each measurement was 10 seconds. Multiple spectra were collected from each sample to avoid an abnormal sample composition.

### 2.4. Data Processing and Analysis

The 1217 spectra of 179 individuals were preprocessed, and all Raman spectral lines were intercepted in the spectral range of 500 cm^−1^-1700 cm^−1^. Due to the instrument, the carrier substrate, the acquired spectra had some background shifts, so noise reduction and debaselining are required. After obtaining the spectrum, first debaseline and denoise each original spectrum using the BEADS algorithm [17], preserving the main peak information and relative intensities. Then, standardize the dispersion of each spectrum (subtract the minimum value of the spectral data and divide it by the form of range), and normalize the spectral data to the range of 0~1 so that all the spectra of each sample occupy the proportion of the following average processing of the same ratio. All spectra for each sample are summed, and dispersion normalized again. That becomes the normalized data for training.

### 2.5. Model Establishment and Verification

A support vector machine (SVM) is a linear binary classifier [18]. Because of the multivariate data set, a one-vs-all multiclass implementation was used to transform this binary classifier into a multiple class discrimination model [19, 20]. In brief, a binary SVM can be extended to distinguish between multiple classes by training an SVM model that all samples in a particular class *y* are labeled as positive, i.e., *c* = +1. Similarly, all other samples are labeled as negative, i.e., *c* = −1; then, finding the class that maximizes the decision function can determine the decision boundary.

Then, a dual-layer cross-validation scheme was used to avoid overestimating and overfitting [21]. In the dual-layer cross-validation, loop data were split into *N* = 5 folds, and each fold as a completely independent test set was used only once. Then, the external training set uses the remaining *N* − 1 folds and splits into *M* = 5 folds in the internal cross-validation loop. Furthermore, data were classified into the internal training data set (*M* − 1 fold) and the validation data set (1 fold) within this inner loop. The internal training set was only used to build the hyperparameter optimization method, and the validation data set was only used to validate, resulting in *M* = 5 validation accuracies. Then, choose the optimal model parameters that show the highest validation accuracy to build the SVM model with the external training set. Lastly, the external training set was used to predict the optimal model. The process is repeated until all the samples are independently tested. Afterward, the testing accuracy is computed using the average of *N* = 5 folds.

## 3. Results

### 3.1. Clinical Features

In the malignant lung cancer group, female patients accounted for 60.3% of the total number of lung cancer patients, the median age was 56, and the range was 32 to 82 years old; pathological stage I accounted for 61.8% of the total lung cancer group. In the benign lung nodule group, female patients accounted for 41.3% of the total benign group, the median age was 53 years, and the range was 23 to 77 years; among normal people, female patients accounted for 53.9% of the normal population, with a median age of 60 years and a range of 25 to 84 years. There was no significant difference in gender (*p* = 0.574) and size (*p* = 0.735) of benign and malignant tumors between groups, and there was no significant difference in tumor location (*p* = 0.707).

### 3.2. Raman Spectroscopy and Statistical Analysis

As shown in Figure 2, there is a certain difference in the mean Raman spectrum of serum between cancer patients and healthy people. Because cancer, benign, and normal people contain a large number of biological macromolecules in the serum, but the content of each biological macromolecule in the serum is different, there is a lot of similar vibration information in the spectrum, but the peak intensity is different. Several representative peaks may involve differences between the sample and control groups. The peaks at 650 cm^−1^ and 857 cm^−1^ represent vibrations of tyrosine, the amount of which increases with cancer progression, while the peak at 734 cm^−1^ may represent vibrations of hypoxanthine. The mean spectra of the benign and malignant groups were almost indistinguishable at the 734 cm^−1^ peaks, indicating that the experimental conditions were practically identical in the two groups. Phenylalanine, a lung cancer biomarker, is located at the peak of 1004 cm^−1^ in the Raman spectrum [22]. Metabolic disorders may cause abnormal content changes of phenylalanine in the lung cancer group. The amide I peak at 1640 cm^−1^, the amide III peak at 1270 cm^−1^, and the tryptophan peak at 1370 cm^−1^ (all of which are higher in cancer patients) have a relatively high average spectral intensity. Raman peaks, such as the uric acid peak at 637 cm^−1^ (higher intensity in cancer patients), also have a certain degree of difference between cancer and benign, indicating that the serum uric acid content is higher in lung cancer patients. This phenomenon may be related to the disorder of purine metabolism in lung cancer patients [23]. Therefore, this shows that it is feasible to use Raman spectroscopy to distinguish benign from malignant.

Figure 2 depicts the mean normalized spectra of the cancer, benign, and normal groups. Aid to appreciate the variability of the data, shaded error bars were meant to indicate one standard deviation from the mean.  Figure 3 depicts the difference spectra, and we can see that spectra from the cancer and benign groups have the most resembling molecular fingerprint. Hence, we hope the classifier mislabels some samples from these groups. However, normal spectra show evident diversity among cancer and benign groups.  Figure 3 shows the 3 groups have an enormous difference in the 734 cm^−1^ bands. The peak at 734 cm^−1^ was assigned to the existence of hypoxanthine. It was found that the SERS intensity of hypoxanthine gradually increases with exposure time because of metabolic degradation in the blood complex [24].

Figure 4 shows the classification results of the support vector machine (SVM) model proposed by us, and the overall accuracy is 93.33%. We can see that only 5 were misclassified and labeled as benign in the 58 cancer samples. And 6 samples were mislabeled, 5 cases were classified as cancer, and 1 case was classified as normal among the 58 benign cases. And there is one sample that was not classified correctly and was given a cancer label in the 63 normal controls. Different spectra show a high error rate between cancer and benign diseases because their molecular fingerprints are highly similar. The ROC curve of the SVM model is shown in Figure 5. The AUC of the three groups (cancer, benign, and normal) is 0.98, 0.97, and 0.99, respectively. These results show that our model has high distinguishing power for cancer.

Table 2 contains the sensitivity, accuracy, and specific values for each category. Our model can specifically distinguish the three groups (i.e., cancer, benign, and the normal). The significant advantage of our classifier is its high sensitivity to normal samples (Se = 0.99). Our two-tier cross-validation and testing of the samples are entirely independent of the samples used in the optimization, ensuring a reliable and repeatable approach that can be extended to real-world clinical settings.

## 4. Discussion

In the development of lung cancer, with the change in metabolic levels in patients, the structure and quantity of many biomacromolecules will also change. SERS can detect the changes in chemical bonds corresponding to these biomacromolecules, so expected to be an effective means of early cancer screening. Early lung cancer screening is still mainly based on low-dose CT. To some extent, a biopsy can help with early diagnosis. However, obtaining bronchoscopy results appeared to be difficult because adenocarcinoma arises in the subsegmental bronchi or alveoli. Such patients generally need an intraoperative biopsy to determine whether the nodules are benign or malignant. Because adenocarcinoma accounts for the majority of pulmonary nodules, the preoperative auxiliary judgment of benign and malignant pulmonary nodules plays an essential role in the clinic that may reduce the risk of excessive medical treatment. From the results of this study, we can see a significant difference between the serum of normal people and patients with benign and malignant pulmonary nodules. The SVM model can predict malignant nodules, benign nodules, and normal with 93.33% accuracy. So the surface-enhanced Raman scattering of serum has great potential in the auxiliary diagnosis of lung adenocarcinoma nodules.

Serum SERS's most crucial detection mechanism is based on enhancing the electromagnetic field caused by the strong localized surface plasmon resonance between the aggregated gold nanoparticles. When the gold colloids are mixed with the serum samples, the biochemical substances in the serum are nonspecifically adsorbed on the surface of gold nanoparticles, resulting in aggregation. And another mechanism involves chemical enhancement caused by charge transfer between the surface of nanoparticles and serum molecules [25, 26]. Due to these two main mechanisms, the Raman signal of the serum can be greatly enhanced, which provides a unique opportunity to explore subtle changes in the serum of patients with early pulmonary nodules at the molecular level.

Compared with normal, the serum SERS signal of the cancer and benign group has some similar changes. The serum samples of malignant and benign pulmonary nodules still contain identical components. The changes in protein-related SERS peaks at 1004 cm^−1^ and 1665 cm^−1^ are usually related to cancer progression and development, which may reflect unique content and conformational changes [27]. And compared with normal controls, a decrease in SERS signal was found at 1004 cm in malignant nodule samples, indicating a reduction in the percentage of phenylalanine and tryptophan relative to the total SERS active components in the blood of cancer patients. The Raman peak at 1004 cm^−1^ is a significant and stable Raman signal that reflects changes in phenylalanine in tissues, cells, blood, and other samples [27].

We know that the peaks at 650 cm^−1^ and 857 cm^−1^ represented the vibration of tyrosine [28], whose content increases as the cancer progresses [29]. And the peak at 734 cm^−1^ represents hypoxanthine [30]. The Raman band near 734 cm^−1^ is the most profound feature among these peaks. However, it was found that the SERS intensity of hypoxanthine gradually diminished with exposure time [31]. Although the dynamic factor will hinder the significance of this band, the approximately zero difference between the benign and malignant groups near 734 cm^−1^ indicates that the sampling condition between these groups was almost identical.

On the other hand, uric acid, xanthine, and hypoxanthine are oxidation products of purine degradation and metabolism in the human body. The metabolic pathway of purine refers to the conversion of hypoxanthine to xanthine and xanthine to uric acid under the action of xanthine oxidase. Therefore, xanthine is the intermediate product of purine metabolism [32]. Xanthine is also an essential biomolecule in the human body. It is a purine base widely distributed in human organs, fluids, and other organisms. It is produced by the catabolism of guanine and adenosine triphosphate in animal muscle tissue. However, its accumulation in the body can lead to death [33]. Prajda's study showed that the imbalance of purine metabolism in liver cancer could be detected. The results showed that xanthine oxidase activity decreased in all liver cancer tissues compared with normal liver tissues, regardless of the tumor's malignant degree, differentiation degree, and growth rate. This phenomenon seems to be specific to the process of tumor genesis [34, 35]. At the same time, compared with normal tissues, the activity of xanthine oxidase in liver cancer is decreased, which reflects the increase in growth rate or different degrees of differentiation. Most importantly, this phenomenon may be the characteristic of tumor proliferation. In addition, the researchers found that xanthine oxidase can inhibit a variety of malignant phenotypes of liver cancer cells and enhance the sensitivity of liver cancer cells to chemotherapeutic drugs.

In addition, because the spectral width at the position of peak 734 cm^−1^ is wide for cancer and benign, and the DNA/RNA base correlation bands (725 cm^−1^,743 cm^−1^) are in this wide range, the intensity is also relatively higher than that of normal people, suggesting that patients with pulmonary nodules may be related to the increase in the relative number of nucleic acid bases relative to the whole active components of SERS. The appearance of these nucleic acid bases may indicate abnormal metabolism of DNA or RNA bases in the blood of patients with pulmonary nodules, which is due to apoptosis and necrosis or the release and lysis of intact cells in the bloodstream. In recent years, the study of circulating RNAs in human blood has attracted much attention because of its role as a new tumor-specific marker in tumor detection [36].

The peak of 1004 cm^−1^ was ascribed to phenylalanine as a biomarker for lung cancer, whose aberrant metabolism may produce content changes [22, 28, 37]. The peaks at 1335 cm^−1^ and 1582 cm^−1^ were found to be tryptophan [28], and its relative SERS intensity was higher in the benign group but decreased in the malignant group, as shown in the previous finding [38, 39]. Although the averaged spectra of the two patient groups differed little, there was still sufficient information which was worth for systematically analyzing.

Currently, surgical diagnosis is recommended for those with solid pulmonary nodules ≥ 8 mm. For the solid pulmonary nodules greater than or equal to 8 mm with a low probability of clinical malignant tumor, the result of functional imaging examination is negative (i.e., the lesion of PET examination does not have hypermetabolism). The test result shows that when the probability of a malignant tumor is very low, the lung nodule cannot be diagnosed by biopsy. As a result, 3-6 months, 9-12 months, or 18-24 months of continuous CT follow-up is recommended. For pulmonary nodules with 6-8 mm diameter, a CT scan is recommended within 6-12 months, and if there is no change, a CT scan is performed within 18-24 months. If the diameter of the pulmonary nodule is 4-6 mm, a CT scan should be performed within 12 months. If there is no change, a subsequent scan is not required. And if the diameter of the pulmonary nodule is less than or equal to 4 mm, no follow-up is needed [40]. Although pulmonary nodules are currently mainly found by CT scan, CT scan cannot determine the benign or malignant nodules. And for nodules of size > 8 mm, expensive PET is needed to further determination, which is difficult for low-income families to bear. Grass-roots hospitals may not have such expensive and complex medical equipment, so patients can only go to higher level hospitals for further examination, making them unable to achieve patient triage. However, blood routine examination equipment is available in every primary medical institution. Raman spectrum screening of serum only needs 2-3 mL blood, which is harmless to the human body, let alone the radiation risk of CT and PET, so the detection based on Raman spectrum screening is a low-cost, easy to carry out screening technology.

It should be noted that the oversimplified peak intensity analysis described above only used limited SERS peak information. At the same time, there are significant changes and overlaps in the SERS spectral intensities of plasma between normal subjects and cancer patients. Therefore, we used multivariate statistical analysis to combine the entire spectrum and automatically determine the most diagnostically essential features to improve serum analysis and differentiation efficiency. Researchers have studied this powerful program to identify Raman spectroscopy in cancer tissues, cells, and blood [41–43]. And our results show that the accuracy of diagnosis of malignant nodules, benign nodules, and normal is 93.33%, which means that lung adenocarcinoma nodules whose pathology cannot be determined before operation can be diagnosed in advance. At present, the positive surgical rate of pulmonary nodules is roughly 80-90%, according to the different levels of different hospitals, which means that some benign patients may receive unnecessary surgery. Our findings suggest that using SERS to identify malignant nodules before an operation is expected to increase by about 10%. From the experimental results, the Raman spectra of benign and malignant nodules are relatively similar, which is also similar to the prediction from a clinical and imaging point of view. For patients with pulmonary nodules, the Raman spectrum is quite different from that of normal people, which indicates that the metabolism of patients with pulmonary nodules is different from that of normal people, which provides a feasible idea for the screening of pulmonary nodules. On the other hand, benign and malignant nodules have similar Raman spectra. This result reflects that the serum components of benign and malignant nodules have similar changes compared with normal, indicating that the samples of pulmonary nodules at different stages still contain some similar components. However, a tumor is a complex system formed in a complex human environment, and it is one-sided to look at a tumor in a single dimension. This study only explored the possibility of an auxiliary diagnosis of benign and malignant pulmonary nodules from the perspective of serum (metabolism/immunity). The AI of imaging has also done a lot of work and feasibility studies from the dimension of imaging. But this paper does not analyze the classification of benign and malignant tumors from the perspective of imaging. So in the next step of work, we will consider continuing in-depth research combining imaging and serum Raman dimensions. One more dimension of information is theoretically helpful for the reliability of auxiliary diagnosis results.

The difference between normal serum and cancer/benign is clear from the results. This shows the sensitivity of this aspect, and the serum can reflect the metabolism and immune status in vivo. Abnormal apoptosis or immunity will lead to certain changes in serum components, and changes in different dimensions reflect the difference between malignant and benign tumors.

This paper uses three groups of variables, normal, benign, and malignant, for statistical analysis, which can accurately classify patients with 93.33% and help detect patients with pulmonary nodules earlier and reduce excessive medical treatment.

## 5. Conclusion

In this work, we prepared gold nanorods as the surface-enhanced Raman spectroscopy detection substrate, which greatly enhanced the Raman signal of serum samples. With the help of the SVM prediction model, our prediction accuracy of malignant nodules, benign nodules, and normal groups reached 93.33%. Our results suggest that surface-enhanced Raman spectroscopy may be fast, effective, and convenient for screening pulmonary adenocarcinoma nodules. It may also provide auxiliary diagnostic information for whether pulmonary nodules should undergo surgery as a reference method for other tumors.

## Figures and Tables

**Figure 1:** Transmission electron microscope image of the synthesized gold nanorods.

**Figure 2:** The average normalized intensity SERS spectra of three groups. The three colored spectra are averaged and normalized spectra with a standard deviation of (a) normal (healthy) group, (b) benign group, and (c) cancer group.

**Figure 3:** The difference between the three groups, (a) cancer vs. benign groups, (b) benign vs. normal groups, and (c) cancer vs. normal groups.

**Figure 4:** The classification results from our proposed SVM model.

**Figure 5:** Receiver-operating characteristic (ROC) curve of SVM model.

**Table 1:** Clinical characteristics of individuals under investigation.

	Cancer (*n* = 58)	Benign (*n* = 58)	Normal (*n* = 63)	*p* value
Type of lung cancer	Adenocarcinoma			
Age, y	57.5 ± 9.6 (32-82)	52.4 ± 11.8 (23-77)	60.4 ± 13.7 (25-84)	0.486
*Sex*				0.574
Male	23	34	26	
Female	35	24	34	
*Pathological stage*				
c-stage IA	28	Nan	Nan	
c-stage IB	15	Nan	Nan	
c-stage IIA	10	Nan	Nan	
c-stage IIB	5	Nan	Nan	
Maximum nodules size, cm	1.55 ± 0.73	1.43 ± 0.6		0.735
*Location*				0.707
Upper lobe of a lung	35	31	Nan	
Middle lobe of a lung	7	7	Nan	
An inferior lobe of a lung	16	20	Nan	

**Table 2:** Performance parameters of the SVM.

Class	Performance parameter	Value ± Std	95% CI
Cancer	Sensitivity	0.92 ± 0.05	0.85-0.98
	Specificity	0.95 ± 0.05	0.89-1.00
	Accuracy	0.94 ± 0.02	0.91-0.96

Benign	Sensitivity	0.92 ± 0.11	0.77-1.00
	Specificity	0.96 ± 0.03	0.92-0.99
	Accuracy	0.94 ± 0.04	0.89-0.98

Normal	Sensitivity	0.98 ± 0.03	0.94-1.00
	Specificity	0.99 ± 0.01	0.96-1.00
	Accuracy	0.98 ± 0.02	0.97-1.00

## Data Availability

The Raman data used to support the findings of this study are available from the corresponding author upon request.
